The article "A Human Torque Teno Virus Encodes a MicroRNA That Inhibits Interferon Signaling" was retracted in 2021. Reasons: results that could not be reproduced; errors in the methods; unreliable data; unreliable images.

# A Human Torque Teno Virus Encodes a MicroRNA That Inhibits Interferon Signaling

**DOI:** 10.1371/journal.ppat.1003818

**Published:** 2013-12-19

**Authors:** Rodney P. Kincaid, James M. Burke, Jennifer C. Cox, Ethel-Michele de Villiers, Christopher S. Sullivan

**Affiliations:** 1 The University of Texas at Austin, Molecular Genetics & Microbiology, Austin, Texas, United States of America; 2 Division for the Characterization of Tumorviruses, Deutsches Krebsforschungszentrum, Heidelberg, Germany; Duke University Medical Center, United States of America

## Abstract

Torque teno viruses (TTVs) are a group of viruses with small, circular DNA genomes. Members of this family are thought to ubiquitously infect humans, although causal disease associations are currently lacking. At present, there is no understanding of how infection with this diverse group of viruses is so prevalent. Using a combined computational and synthetic approach, we predict and identify miRNA-coding regions in diverse human TTVs and provide evidence for TTV miRNA production *in vivo*. The TTV miRNAs are transcribed by RNA polymerase II, processed by Drosha and Dicer, and are active in RISC. A TTV mutant defective for miRNA production replicates as well as wild type virus genome; demonstrating that the TTV miRNA is dispensable for genome replication in a cell culture model. We demonstrate that a recombinant TTV genome is capable of expressing an exogenous miRNA, indicating the potential utility of TTV as a small RNA vector. Gene expression profiling of host cells identifies N-myc (and STAT) interactor (NMI) as a target of a TTV miRNA. NMI transcripts are directly regulated through a binding site in the 3′UTR. SiRNA knockdown of NMI contributes to a decreased response to interferon signaling. Consistent with this, we show that a TTV miRNA mediates a decreased response to IFN and increased cellular proliferation in the presence of IFN. Thus, we add Annelloviridae to the growing list of virus families that encode miRNAs, and suggest that miRNA-mediated immune evasion can contribute to the pervasiveness associated with some of these viruses.

## Author Summary

The torque teno viruses (TTVs) are a diverse group of viruses that ubiquitously infect humans and establish persistent infections. Despite their prevalence, TTVs lack concrete disease associations and remain among the most poorly characterized human viruses. Here we use computational and synthetic approaches to identify new noncoding miRNA genes in the TTVs. We demonstrate that TTVs utilize the host miRNA biogenesis machinery to produce biologically active miRNAs. To gain a functional understanding of the new TTV genes, we focus on a particular viral isolate and identify N-myc (and STAT) interactor (NMI) as a direct target. NMI is a known modulator of interferon and cytokine signaling. Similar to other viruses encoding miRNAs, the TTVs likely utilize miRNAs to promote persistence and immune evasion. Our study provides new insights into novel TTV gene products and the interactions of this virus with its host.

## Introduction

Torque teno viruses (TTVs) belong to the family *Anelloviridae* and have small (∼3.8 kb) circular, ssDNA genomes [1]. While these viruses are compact in their genomic size, there is a surprising amount of diversity reported in viral isolates, and the human TTVs have been phylogenetically classified into five groups [2]–[4]. The first TTV like sequence was isolated from a patient with non-A–G hepatitis [5]; however, TTVs are not currently thought to have a causal role in such disease and no concrete disease associations currently exist [6]. Despite the current lack of clear disease associations, TTVs are considered near ubiquitous in the human population and appear to establish persistent infections in their host [6]. Exactly how TTVs are able to evade clearance by the host immune response and establish long term persistent infections remains a mystery which solving may require the identification of the full complement of TTV gene products and their functions.

MicroRNAs (miRNAs) are small ∼22 nt noncoding RNAs that direct posttranscriptional gene regulation. miRNAs were first identified in the nematode *C. elegans* [7], but since have been recognized as important regulators of gene expression in many eukaryotes and even viruses [8]. Diverse viruses including some members from the Herpesvirus, Polyomavirus, and Retrovirus families have been confirmed to encode viral miRNAs [9]. While these virus families are different in many ways, they do share some commonalities including a nuclear DNA component to their replicative cycle and the ability to establish persistent infections in their hosts. Emerging themes of viral miRNA function include immune evasion, prolonging longevity of host cells, and regulation of persistent versus productive infection [9]–[11]. Unlike most protein-based viral gene products, viral miRNAs are thought to be relatively invisible to the host immune system [8] and require minimal genomic space for their encoding.

The extent to which different virus families utilize miRNAs remains a fundamental question in the field of viral miRNAs. To address this question we have previously developed computational methods to predict miRNA genes from primary sequence information [12]. Using this approach as a starting point, we investigated the TTV family for the potential to encode miRNAs. A diverse group of viral miRNAs encoded by TTVs were identified and their interactions with the host miRNA biogenesis pathway characterized. We have generated recombinant TTVs capable of expressing a small RNA transgene as well as a miRNA mutant virus to study miRNA function. Gene expression profiling led to the discovery of a direct target of a TTV miRNA, N-myc (and STAT) interactor (NMI). NMI is an interferon stimulated gene known to modulate interferon and cytokine signaling [13] and has been previously associated with viral induced apoptosis [14]. Furthermore, we demonstrate an inhibitory role for a TTV miRNA in interferon signaling. Our findings support the model that TTVs make use of viral miRNAs to modulate the innate immune response and promote their persistence.

## Results

### A Combined Computational and Synthetic Approach Identifies TTV Encoded miRNAs

We investigated TTV genomic sequences for miRNA gene candidates using previously described computational methods that predict candidate pre-miRNAs [12]. Since most miRNAs are not coded within protein coding sequences, our search for predicted miRNA candidates focused on regions of the viral genomes lacking protein coding sequence annotation. This restriction has the added advantage of significantly reducing the search space. Candidate pre-miRNA sequences in multiple human TTVs were observed within an unannotated region between the poly A signal of the known viral transcripts and the canonical promoter region (Figure 1A, Table S1). Some TTV strains had a single pre-miRNA-like stemloop prediction, while other strains had two pre-miRNA-like stemloop predictions in this region (Figure 1A). We therefore chose to test predictions from both classes. The candidate viral pre-miRNA sequences were commercially synthesized and tested by transfection of HEK293T cells followed by Northern blot analysis. This revealed readily detectable signals migrating at the appropriate sizes that corresponded to the predicted derivative miRNA sequences (Figures 1B, 1D). Based on these results, promising candidates were also subjected to high throughput small RNA sequencing to look for features common to bona fide miRNAs. The small RNA sequencing libraries contained small RNA reads that mapped specifically to the predicted pre-miRNA sequences (Figures 1C, 1E). Importantly, these small RNAs displayed the features expected of true miRNAs– predominant derivatives arising from each arm of the stem loop structure and predicted 3′ ∼2 nucleotide overhangs (Figure 1A). Taken together, these results strongly support the production of miRNAs from the computationally predicted, synthetic constructs.

**Figure 1:** A combined computational and synthetic approach identifies TTV encoded miRNAs. (A) Diagram of genomic locations of predicted TTV-yonKC197 (AB038624) and TTV-TWH (AFL351132) miRNAs. Reference sequence annotated ORFs are indicated in red and predicted miRNA stemloop sequences are indicated in blue. Secondary structure predictions of the putative TTV miRNAs are shown to the right with bolded sequences indicating most abundant mature miRNA sequences observed in small RNA sequencing library. (B) Northern blot analysis of RNA harvested from HEK293T cells transfected with synthetic TTV-yonKC197 miRNA vector (SG for “synthetic gene”) or empty vector (NC). Ethidium bromide stained low molecular weight RNA is shown as a load control. (C) Northern blot analysis of RNA harvested from HEK293T cells transfected with synthetic TTV-TWH miRNA vector (SG) or empty vector (NC). Ethidium bromide stained low molecular weight RNA is shown as a load control. (D) Pooled small RNA profiling of HEK293T cells transfected with TTV-yonKC197 miRNA vector. Sequences were mapped to the synthetic region of the AB038624 NCBI reference sequence. The vertical axis depicts small RNA read coverage observed; while the horizontal axis shows the relative position within the synthetic gene sequence. (E) Pooled small RNA profiling of HEK293T cells transfected with TTV-TWH miRNA vector. Sequences were mapped to the synthetic region of the AFL351132 NCBI reference sequence. The vertical axis depicts small RNA read coverage observed; while the horizontal axis shows the relative position within the synthetic gene sequence.

Next, we asked whether TTV derived miRNAs are detectable during viral replication. We chose to utilize a previously described cell culture based replication system using the TTV-tth8 strain [4], [15]. The TTV-tth8 strain has one predicted miRNA stemloop located in the non-coding region (NCR) (Figure 2A). Northern blot analysis was performed on total RNA extracted from the replication system as well as from HEK293T cells transfected with a synthetic vector containing the predicted miRNA sequence (Figure 2B). Similar signals consistent with detection of both the pre-miRNA and a mature miRNA were observed from both our synthetic construct and the viral replication system. These data confirm that TTV-encoded miRNAs are produced during replication of the TTV-tth8 genome in cell culture.

**Figure 2:** TTV miRNAs are expressed during *in vitro* cell culture replication and are detectable from *in vivo* small RNA profiling of human PBMCs. (A) Diagram of genomic locations of predicted TTV-tth8 (AJ260231) miRNA. Reference sequence annotated ORFS are indicated in red and predicted miRNA stemloop sequence is indicated in blue. Secondary structure prediction of the putative TTV miRNA is shown below with bolded sequences indicating most abundant mature miRNA sequences observed in small RNA sequencing library. (B) Northern blot analysis of RNA harvested from HEK293T cells transfected with synthetic TTV-tth8 miRNA vector (SG) or empty vector (NC) and HEK293TT cells transfected with viral genome prep (TTV) or mock transfection (Mock). Northern blot analysis for host miRNA hsa-miR-19a and ethidium bromide stained low molecular weight RNA serve as load controls. (C) Small RNA profiling of human PBMC small RNAs mapped to TTV-sle2057 strain. The vertical axis depicts small RNA read coverage observed; while the horizontal axis shows the relative position within the TTV-sle2057 genomic sequence.

To determine whether TTV viral miRNAs are expressed *in vivo*, small RNA libraries deposited in the NCBI Sequence Read Archive (SRA) were examined [16]. A data set deposited by Vaz *et al* included two small RNA sequencing libraries derived from primary human PBMCs from apparently healthy individuals [17]. These small RNA libraries were mapped to a collection of deposited TTV and TTV-like viral genomes (Table S2). Of the two samples we examined, one of the libraries (SRR039191) contained reads mapping specifically to predicted miRNA stemloop structures of TTV-sle2057 and related strains (Figure 2C). While the total number of reads mapped to TTV miRNAs was low, this might be expected since only a small fraction of the PBMC population would be expected to harbor the virus and the total number of reads sequenced was relatively small (∼3 million total reads). Furthermore, the fact that the reads mapped only to the exact miRNA predicted structures and not elsewhere in the viral genome or the human genome, strongly supports the sequences being of viral origin. Thus, we conclude that TTV-encoded miRNAs are expressed in their human hosts during infection.

### Diversity of Anellovirus Encoded miRNAs

The Anellovirus family includes the torque teno viruses (TTVs), torque teno midi viruses (TTMDVs), torque teno mini viruses (TTMVs), as well as related nonhuman animal viruses [2]. The TTMDVs and TTMVs share similar genomic organization with TTV but have significantly shorter genomic sequences. A computational based search for predicted miRNA-like sequences was carried out on deposited TTV and the related TTMDV and TTMV genomic sequences (Table S1). No strong miRNA candidates were identified from either the TTMDVs or TTMVs (data not shown). It is worth noting that many of the deposited TTMDV and TTMV sequences have a much shorter NCR than TTVs. This observation may in large part be due to the incomplete nature of some submitted viral genomic sequences. While our initial bioinformatics strategy failed to identify likely candidates in these sequences we cannot rule out the possibility they were missed by our bioinformatics analysis or due to a lack of verified full length genomic sequences.

### TTV tth8 miRNA Is Processed by the Canonical Host miRNA Pathway

The majority of known human and viral miRNAs follow a canonical biogenesis pathway that begins with transcription by host RNA polymerase II. The pri-miRNA transcript is cleaved by the enzyme Drosha, which is the nuclease component of the Microprocessor complex, to liberate the short stem loop pre-miRNA [18]. The pre-miRNA may then be exported to the cytoplasm whereupon it is cleaved by a second nuclease, Dicer, to generate a short ∼22 nt duplex RNA [19]. Typically, one strand of this duplex RNA is loaded into the RNA Induced Silencing Complex (RISC) where it may direct RISC mediated repression to target RNAs [20]. While most host miRNAs and viral miRNAs utilize this common pathway, notable exceptions have been reported from both the herpesvirus and retrovirus families [12], [21], [22].

Our miRNA biogenesis and functional characterization focused on TTV isolate tth8 (TTV-tth8) due to the availability of an *in vitro* cell culture virus genome replication system [4], [15]. We began by investigating the mode of transcription. Treatment of cells with an appropriate concentration of α-amanitin inhibits RNA polymerase II transcription but not transcription by RNA polymerase III [21]. HEK293 cells were transfected with re-circularized TTV tth8 viral genome in the presence or absence of α-amanitin and then miRNA expression was assayed by Northern blot. As controls, a recombinant TTV expressing the SV40-miR-S1 miRNA– an RNA pol II dependent miRNA, or vector encoding the RNA pol III-transcribed miRNA MHV68-miR-M1-7 were also tested. As shown in Figure 3A, the expression of the positive control SV40-miR-S1 and TTV-tth8-miR-T1 miRNAs are both inhibited by α-amanitin, while as expected, the negative control pol III-dependent MHV68-miR-M1-7 miRNA was resistant to treatment. In addition, we observed similar results when transfecting HEK293T cells with vectors containing our synthetic TTV miRNA candidates (Figure S1A). These data are consistent with the TTV miRNAs being derived from RNA pol II transcripts, similar to most previously described host and viral miRNAs.

**Figure 3:** TTV tth8 miRNAs are generated by the canonical host miRNA biogenesis pathway. (A) Northern blot analysis of RNA from HEK293 cells transfected with MHV68-miR-M1-7 expression vector, SV40-miR-S1 TTV recombinant genome preparation, or wildtype TTV-tth8 genome preparation with or without treatment with the RNA pol II inhibitor α-amanitin. Ethidium bromide stained low molecular weight RNA is shown as a load control. (B) Northern blot analysis of RNA from HEK293T cells co-transfected with MHV68-miR-M1-7, SV40-miR-S1, or TTV-tth8-miR-T1 expression vectors and either Drosha siRNA (siDrosha) or negative control siRNA (siNC). Ethidium bromide stained low molecular weight RNA is shown as a load control. (C) Northern blot analysis of RNA from either DLD1 (WT) or DLD1DicerEx5- (DicerEx5-) cells transfected with either MHV68-miR-M1-7 or TTV-tth8-miR-T1 expression vectors. Ethidium bromide stained low molecular weight RNA is shown as a load control. (D) RISC reporter assay for TTV-tth8-miR-T1. HEK293 cells were co-transfected with either empty miRNA expression vector (Vector) or TTV-tth8-miR-T1 expression vector (TTH8) and both control firefly luciferase reporter and *Renilla* luciferase based reporter plasmids with vector UTR (Vector), two sites perfectly complementary to TTV-tth8-miR-T1-5p (5p), two sites perfectly complementary to TTV-tth8-miR-T1-3p (3p), or control 3′UTR reporter with GAPDH 3′UTR (GAPDH). The average relative *Renilla* luciferase activity normalized to firefly luciferase activity of three replicates is shown. Error bars indicate SD of three replicates and p-values were calculated using Student's t-test.

Next, we investigated the role of Drosha, the endonuclease component of the Microprocessor responsible for excising pre-miRNAs from pri-miRNA transcripts. HEK293Tcells were transfected with siRNA directed against Drosha [23] (or negative control siRNAs) followed by transfection of miRNA expression vectors and Northern blot analysis. Drosha-dependent SV40-miR-S1 miRNA, or the Drosha-independent MHV68-miR-M1-7 miRNA expression vectors, were used as controls. As expected, the Drosha siRNA treatment inhibited expression of the SV40-miR-S1 miRNA, but did not have a significant effect on the expression of the MHV68-miR-M1-7 miRNA (Figure 3B). The effect of the Drosha siRNA treatment with the TTV-tth8-miR-T1 expression vector was similar to the SV40-miR-S1 miRNA. Furthermore, similar results were observed when transfecting HEK293T cells with vectors containing our synthetic TTV miRNA candidates (Figure S1B). Therefore, we conclude that the TTV miRNAs are processed in a Drosha-dependent manner similar to most previously described host and viral miRNAs.

Dicer is the endonuclease responsible for processing pre-miRNAs into mature miRNA duplex RNAs. DLD1-DicerEx5- is a Dicer-activity-hypomorphic cell line which exhibits impaired conversion of pre-miRNAs to mature miRNAs [24]. This defect results in decreased Dicer-processed mature miRNA production and an accumulation of pre-miRNA substrate. TTV-tth8-miR-T1, or the positive control Dicer-dependent MHV68-miR-M1-7 miRNA expression vectors, were transfected into the Dicer hypomorph or isogenic wild type Dicer parental cell lines and then assayed by Northern blot (Figure 3C). Like the MHV68-miR-M1-7 control, a pre-miRNA:miRNA ratio change consistent with Dicer processing was observed with TTV-tth8-miR-T1. Thus, we conclude that the TTV-tth8 miRNAs are processed in a Dicer-dependent manner similar to most previously described host and viral miRNAs.

The final step in the canonical miRNA biogenesis pathway is the incorporation of the mature miRNA into active RISC. Luciferase based reporter constructs specific to each arm of TTV-tth8-miR-T1 miRNA were generated to test for RISC activity. The luciferase based reporter constructs were co-transfected with a TTV-tth8-miR-T1 miRNA expression vector, or control vector, and then dual luciferase assays were performed (Figure 3D). The relative expression of either TTV-tth8 reporter construct was significantly inhibited by co-transfection of the TTV-tth8-miR-T1 expression vector, while no significant difference was observed with either of two negative controls– vector 3′UTR or an irrelevant GAPDH 3′UTR reporter. Similar results were observed with our synthetic TTV miRNA candidates and corresponding reporter constructs (Figure S1C). Therefore, we conclude that the TTV miRNAs are active in RISC.

Taken together, we have identified the general pathway through which biologically active miRNAs are generated. The evidence presented is most consistent with direct utilization of the canonical host miRNA biogenesis machinery.

### Generation and Characterization of Recombinant TTVs

A mutant TTV-tth8 with ablated miRNA production (TTV-MUT) was generated by introduction of a specific 4 nt deletion into the miRNA stem region (Figure 4A). A recombinant TTV was generated by inserting the SV40-miR-S1 sequence into the same genomic position. Generation of this TTV-SV40 recombinant virus (TTV-SV40) serves two purposes: (1) As an additional control in our functional analysis and, (2) As an initial test of the TTV as a potential small RNA vector. HEK293TT cells were transfected with circularized viral genome preparations and assayed for miRNA expression by Northern blot analysis (Figure 4B). As expected, we were unable to detect production of the TTV-tth8-miR-T1 from TTV-MUT or TTV-SV40. However, we were able to detect the production of the SV40-miR-S1 from TTV-SV40 recombinant as anticipated. Thus, we have successfully generated a surgical miRNA mutant virus and have demonstrated the capacity of the TTV-tth8 virus to express an exogenous miRNA.

**Figure 4:** Generation of mutant and SV40 recombinant TTVs. (A) RNA secondary structure predictions of miRNA region from TTV-tth8 wildtype, TTV-tth8 miRNA mutant, and TTV-tth8 SV40 recombinant viruses. (B) Northern blot analysis of total RNA harvested from HEK293TT cells transfected with either pUC plasmid (Vector), wildtype TTV-tth8 (TTH8 WT), miRNA mutant TTV-tth8 (TTH8 MUT), or SV40 miRNA recombinant TTV-tth8 (TTH8 SV40). Northern blot analysis for host miRNA hsa-miR-19a and ethidium bromide stained low molecular weight RNA serve as load controls.

While we have shown that TTV-MUT does not produce TTV-tth8-miR-T1, it was still possible that other miRNAs could be encoded by the virus that our prediction methods missed. To address this concern and better characterize the miRNAs encoded by TTV-tth8, high throughput small RNA sequencing was performed on small RNA fractions harvested from the cell culture replication system for both the wildtype TTV-tth8 and TTV-MUT (Figure 5). As expected, abundant small RNA reads mapping to TTV-tth8-miR-T1 were observed for the wildtype virus but not TTV-MUT. Interestingly, a lesser amount of antisense mapping reads were observed for TTV-tth8-miR-T1, which would be indicative of transcription and specific processing of the antisense strand as well. We note that it has previously been reported that TTV replication generates antisense transcripts of unknown function [15]. However, no pattern of reads indicative of miRNA production was observed from TTV-MUT or additional outside of the TTV-tth8-miR-T1 locus in the wildtype virus. Therefore, we conclude that TTV-tth8 encodes miRNAs at a single locus and we have successfully generated a miRNA null variant.

**Figure 5:** Characterization of wildtype and miRNA mutant TTV-tth8. Small RNA profiling of HEK293TT cells transfected with either wildtype TTV-tth8 (WT) or miRNA mutant TTV-tth8 (MUT). At top, ORF map derived from NCBI reference sequence AJ260231 annotations in red. The newly identified miRNA is indicated in blue. The vertical axis depicts small RNA read coverage observed; while the horizontal axis shows the relative position within the TTV-tth8 genomic sequence.

We hypothesized that the disruption of TTV-tth8-miR-T1 would alter viral replication dynamics. To test this hypothesis, timecourse experiments were performed with TTV-tth8 and TTV-MUT in the cell culture replication system. DpnI protection assays were performed to differentiate between replicated and non-replicated viral DNA [4], [25]. DpnI is a restriction endonuclease that recognizes only a methylated form of the restriction site. The viral genomic DNA prepared from bacterial stocks is methylated while viral DNA that is replicated in the HEK293TT cells will not be methylated at the restriction site. DpnI protection assays followed by Southern blot analysis were performed on DNA harvested at timepoints up to 9 days post initial transfection (Figure S2). We did not observe any gross differences in viral genome replication between the wildtype (WT) and mutant (MUT) viruses in this assay. However, we note that similar lack of cell culture replication defects have been reported for some miRNA mutant viruses from the polyoma and herpes families in cell culture [26], [27], and that this result does not rule out the possibility for replication differences *in vivo*.

### Identification of TTV-tth8-miR-T1 Targets by Microarray Analysis

Programming of RISC with a mature miRNA sequence directs the complex to target mRNAs resulting in translational repression and enhanced turnover of some of the target mRNAs [28], [29]. The enhanced turnover of target mRNAs can result in lower steady state transcript levels that can be detected via microarray analysis [30]–[34]. As a preliminary investigation of possible host targets for TTV-tth8-miR-T1, microarray analysis for human transcripts was performed on RNA harvested from HEK293TT cells transfected with TTV-tth8, TTV-MUT, TTV-SV40, or pUC control vector. To identify candidate direct targets, the following criteria were applied: putative targets must be lower in the wildtype sample than the mutant or SV40 control and a seed complementary sequence must be present in the 3′UTR sequence of the candidate. Using this approach, 16 candidates were identified that were differentially expressed between the samples and that possessed seed complementary sequences in their 3′UTRs (Table S3). We caution that such analysis should be used for preliminary hypothesis generation, and subsequent confirmation experiments are required to establish direct effects. Examining the list for candidates with known functions in viral infection led us to the gene N-myc (and STAT) interactor (NMI). As an interferon stimulated gene (ISG) [35], a regulator of STAT signaling [13], and because of its involvement in virus-induced apoptosis [14], we chose to further investigate this putative target.

### NMI Is a Direct Target of TTV-tth8-miR-T1

We identified a putative miRNA binding site for the more abundant 5p arm of TTV-tth8-miR-T1 in the 3′UTR of NMI (Figure 6A). To test whether TTV-tth8-miR-T1 can directly target this sequence, luciferase reporter constructs with the full length NMI 3′UTR as well as a reporter construct with the full length NMI 3′UTR with a 2 nt change in the predicted seed docking site were generated. HEK293T cells were co-transfected with the luciferase based reporter constructs and a TTV-tth8-miR-T1 miRNA expression vector, SV40-miR-S1 vector, or control vector and dual luciferase assays were performed (Figure 6B). The relative expression of the NMI 3′UTR reporter construct was significantly inhibited by co-transfection of the TTV-tth8-miR-T1 expression vector while no significant difference was observed with vector 3′UTR control or an irrelevant GAPDH 3′UTR reporter control. Importantly, no significant difference was observed when the seed mutant 3′UTR reporter was co-transfected with the tth8-miR-T1 expression vector, which strongly supports that the regulation observed is through docking at our predicted miRNA target site.

**Figure 6:** Host antiviral gene NMI is a direct target of TTV-tth8-miR-T1. (A) Diagram of predicted TTV-tth8-miR-T1-5p docking site in the 3′UTR of NMI transcripts (top) with complementary base pairing to the TTV-tth8-miR-T1-5p (middle) seed indicated (“|” for predicted base pairing and “·” for wobble pairing). At bottom is diagrammed the seed mutant (NMI MUT) sequence with the introduced two nucleotide mismatch in the seed complementary region (underlined sequence). (B) NMI 3′UTR miRNA docking site reporter assay. HEK293 cells were co-transfected with either empty miRNA expression vector (Vector), TTV-tth8-miR-T1 expression vector (TTH8), or SV40-miR-S1 expression vector (SV40) and both control firefly luciferase control and *Renilla* luciferase based reporter plasmids with vector UTR (Vector), full length NMI 3′UTR (NMI), full length NMI 3′UTR with 2 nt mutation in predicted docking site (NMI MUT), or control 3′UTR reporter with GAPDH 3′UTR (GAPDH). The average relative *Renilla* luciferase activity normalized to firefly luciferase activity of three replicates is shown. Error bars indicate SD of three replicates and p-values were calculated using Student's t-test. (C) Immunoblot analysis of total protein harvested from HeLa cells transfected with either TTV-tth8-miR-T1 miRNA mimic (miTTH8) or negative control miRNA mimic (miNC). Shown is a representative blot. (D) Quantification of the average of three independent experiments as in panel C. Error bars indicate SD of three independent experiments and p-values were calculated using Student's t-test.

While TTV-tth8-miR-T1 can directly regulate reporter constructs bearing the NMI 3′UTR, we next wanted to know if TTV-tth8-miR-T1 can regulate expression of NMI protein from endogenous NMI transcripts. A miRNA mimic of TTV-tth8-miR-T1 was synthesized based on the sequences from our small RNA profiling experiments. HeLa cells were transfected with the viral miRNA mimic or negative control miRNA mimic and NMI protein levels were assayed by immunoblot analysis (Figure 6C). A modest but highly reproducible decrease in NMI protein levels (∼25%) with TTV-tth8-miR-T1 mimic transfection was observed in three independent experiments (Figure 6D). Therefore, we conclude that NMI is a direct target of TTV-tth8-miR-T1.

### TTV-tth8-miR-T1 miRNA Mimic or siRNA Targeting NMI Inhibits Interferon Signaling

NMI has previously been shown to modulate STAT signaling pathways in response to cytokine stimulation. A luciferase based interferon signaling assay was employed to determine whether TTV-tth8-miR-T1 can modulate interferon signaling activity (Figure 7A). Dual luciferase assays were performed on HEK293T cells co-transfected with circularized viral genomes or control plasmid and luciferase reporters and subsequently treated with universal type I interferon (Figure 7B). Relative to control plasmid, a ∼40% decrease in ISRE driven luciferase activity was observed with wildtype TTV-tth8 while a ∼18% decrease was observed with the miRNA mutant TTV-tth8. Although additional viral factors may contribute to the decreased activity in this assay, a significantly larger decrease was observed with the miRNA competent virus.

**Figure 7:** TTV-tth8-miR-T1 or knockdown of NMI inhibits interferon signaling. (A) Schematic of the interferon signaling assay. Target cells are co-transfected with dual luciferase plasmids (firefly luciferase with interferon-stimulated response element (ISRE) based promoter and transfections control Renilla luciferase with constitutive promoter) and either re-circularized viral genome, miRNA mimic, or siRNA. Forty-eight hours later, cells are treated with 100 U/mL Type I interferon. Sixteen hours after interferon treatment, dual luciferase assay is performed. (B) Interferon signaling assay performed as outlined in Fig. 7A with TTV-tth8 wildtype (WT) and miRNA mutant (MUT) genomic preparations in HEK293T cells. Relative luciferase activity is normalized to pUC19 vector control (VEC). Error bars indicate SD of three replicates and p-values were calculated using Student's t-test. (C) Interferon signaling assay performed as outlined in Fig. 7A with miRNA mimics and siRNAs in HEK293T cells. TTV-tth8 miRNA mimic (miTTH8) was normalized to negative control miRNA mimic (miNC). NMI siRNA was normalized to negative control siRNA (siNC). Co-transfection of both a miRNA mimic and siRNA is indicated by a “/” and was normalized to co-transfection of both siNC and miNC. Error bars indicate SD of three replicates and p-values were calculated using Student's t-test. Not significant (n.s.) indicates p-value greater than 0.05. (D) Interferon signaling assay performed as outlined in Fig. 7A with miRNA mimics in HEK293T and ISG15 expression assayed by qPCR following interferon treatment. TTV-tth8 miRNA mimic (miTTH8) treatment was normalized to negative control miRNA mimic (miNC). NMI siRNA (siNMI) treatment was normalized to negative control siRNA (siNC). Relative ISG15 expression was determined by comparative Ct method to GAPDH. Error bars indicate SD of three replicates and p-values were calculated using Student's t-test. (E) Growth curves of interferon treated B cell lines that stably overexpress the TTV tth8 miRNA (TTH8) or a negative control irrelevant miRNA (NC) or vector alone (VEC). Viable cells as determined by trypan blue staining were counted each day and then either mock-treated with BSA or treated with universal type I IFN (+IFN). Data points represent averages of three independent experiments (each performed in triplicate) on different days and error bars indicate SD of the three experiments.

To further investigate the effects of TTV-tth8-miR-T1 and NMI on interferon signaling, interferon reporter assays were performed with synthetic miRNA mimics or siRNA directed against NMI (Figures 7C, S3). Relative to control mimic, transfection of HEK293T cells with the TTV-tth8-miR-T1 mimic resulted in a significant reduction in expression of the ISRE driven reporter (∼50%) (Figure 7C). Transfection of siRNA targeted against NMI resulted in a similar reduction in reporter expression. However, co-transfection of both siRNA against NMI and TTV-tth8-miR-T1 mimic did not exhibit an additive effect. Similar results were observed in experiments conducted in HeLa cells (Figure S3B). To determine if the interferon reporter assays were reflective of endogenous ISRE activity, quantitative Real-Time PCR (qRT-PCR) for an endogenous ISG transcript (ISG15) was performed on RNA extracted from HEK293T cells treated with interferon (Figure 7D). Relative ISG15 levels were significantly reduced (∼40%) with transfection of either TTV-tth8 miRNA mimic or NMI siRNA with respect to negative control miRNA mimic or siRNA. These results provide support that the luciferase-based ISRE reporter system is reflective of endogenous ISRE activity. Although we cannot rule out that additional targets of TTV-tth8-miR-T1 contributed to the decreased reporter activity, the evidence presented suggests that targeting of NMI by TTV-tth8-miR-T1 contributes to decreased interferon signaling.

Finally, we examined the effects of TTV-tth8 miRNA expression on cells exposed to interferon. We chose a low passage PBMC-derived human B-cell line since PBMCs likely serve as host cells to TTVs *in vivo* (reviewed in [6]). Pooled stable cell lines expressing either the TTV-tth8 miRNA, an irrelevant control miRNA, or vector were generated by lentiviral transduction of human B-cell line GM19240. Growth curves were calculated for all three cell lines in the presence or absence of interferon (Figure 7E). All three cell lines grew similarly in the absence of interferon. Treatment with daily interferon resulted in a marked defect in growth in both controls cell lines (vector alone and irrelevant miRNA). In contrast, in the presence of IFN treatment, the TTV-tth8 miRNA-expressing cell line exhibited ∼10 fold more viable cells (compared to the control cell lines) at the conclusion of the growth curve. Therefore, we conclude that the TTV-tth8 miRNA can promote cell growth/viability under some interferon-rich conditions.

## Discussion

Although the first viral miRNAs were reported over nine years ago [36], a comprehensive understanding of which virus families encode miRNAs remains incomplete. In this study we have added another family, *Anelloviridae*, to the growing list of virus families with members encoding miRNAs. This is the first ssDNA virus reported to encode miRNAs. The TTVs remain among the most poorly studied of human viruses, perhaps due to a lack of conclusive disease associations. However, the ability of TTVs to establish ubiquitous persistent infections implies that studying the TTVs can reveal important lessons in viral persistence that may be useful in understanding other virus families as well.

The mechanisms by which TTVs are able to establish persistent infections and avoid clearance by the immune system remain elusive. In this study we have demonstrated that some TTVs encode miRNAs which are thought to be non-immunogenic regulatory molecules. We hypothesized that TTVs may utilize these effectors to target transcripts of their host cell. We identified a direct target of TTV-tth8-miR-T1, NMI. NMI is a transcription cofactor that can modulate the activity of members of the STAT family in response to interferon and cytokine signaling [13]. Recently, NMI has been implicated in additional roles including: inhibition of Wnt/β-catenin signaling [37], tumor suppressive activity when exogenously expressed in a mouse tumor model [37], and protection of the tumor suppressor ARF from degradation during stress [38]. While our current results support the idea that TTV-tth8 miRNA targets NMI to inhibit interferon signaling and promote immune evasion, NMI may not be the only, or even the major target responsible for the effects of the TTV-tth8 miRNA that we observe. Furthermore, it is likely that other functions for the TTV-tth8 miRNA are possible. However, the observation that expression of the TTV-tth8 miRNA in B-cell lines provides partial resistance to interferon-induced growth defects provides additional support for an immune evasion role for this miRNA. Thus, it is likely that some TTVs, similar to other viruses encoding miRNAs [9], [10], utilize miRNAs in immune evasion and to promote their persistence.

Do the TTV encoded miRNAs serve additional noncanonical functions? While we have focused on possible canonical miRNA functional roles, we cannot rule out that the TTV miRNAs may provide additional functional benefits to the virus. For example, we observe that the TTV miRNAs are encoded proximal to the major poly A site for the protein coding viral transcripts, and a similar arrangement is observed in the polyomaviruses SV40, JCV, and BKV in which the viral miRNAs are encoded proximal to the poly A site for the late transcripts [26], [39]. We hypothesize that the presence of stemloop structures could provide additional benefits including the imposition of greater transcriptional termination of the mRNAs which could be of benefit to viruses with small circular genomes. Furthermore, we observed evidence that TTV-tth8 transcripts in both orientations over the miRNA locus are subject to post-transcriptional cleavage (Fig. 5A). It is tempting to speculate that this phenomenon could provide benefit to a small circular virus in the prevention of the accumulation of double stranded RNA (dsRNA), a potential pathogen associated molecular pattern [40].

TTVs with human hosts have been noted for their great genetic diversity despite their limited coding capacity [41]. Here we identified a new genetic locus encoding miRNAs. Perhaps not surprisingly, TTVs display significant diversity at this newly identified locus as well. The TTVs and their diversity are a ripe area for future evolutionary studies to understand how viral miRNAs, and noncoding RNAs in general, evolve and how they influence viral diversity. Strong miRNA candidates were observed from all five groups of human TTVs as well as some related primate TTVs (Table S1). However, no strong miRNA candidates were observed in the related TTMDVs or TTMVs (data not shown). It is worth noting that deposited sequences of both of these groups of viruses have shorter NCRs which in some part may be due to the submission of incomplete viral genomic sequences. It is also possible that some of these viruses lack miRNA genes and may have evolved alternative strategies to fulfill any beneficial roles of the TTV miRNAs. Furthermore, we did not observe strong miRNA candidates from various non-primate TTVs at the same locus, but there are relatively few full length reported strains for most of the TTVs with non-human hosts. Future studies and sequencing of additional isolates will be needed to address the roles, if any, of miRNAs in the non-human TTVs and related anelloviruses.

Can TTVs be harnessed as potential therapeutic vectors? An attractive quality of TTV is the implied low pathogenicity of TTVs from lack of strong disease associations and their ubiquitous nature. Average TTV titers of 10∧4 to 10∧6 genome copies per mL of blood have been reported for apparently healthy individuals [42], [43]. While the TTV genome itself has limited coding capacity for transgenes, we have demonstrated that exogenous small RNAs can be expressed from the viral genome (Fig. 4B). However, current attempts to vectorize the TTVs may be limited by lack of fundamental knowledge of TTV biology and limited culture systems. While the possible use of TTV as a small RNA vector awaits a more complete understanding of the replication and life cycle of these viruses, our work at least establishes the ability of these genomes to readily express a heterologous miRNA.

In summary, we have demonstrated that a ubiquitous human virus encodes novel miRNAs, one of which may antagonize the host antiviral response. Our findings bring new insights into the torque teno viruses as well as their interactions with the host miRNA machinery and antiviral response.

## Methods

### Cell Lines

HeLa, HEK293, and HEK293T obtained from American Type Culture Collection (ATCC) were maintained in DMEM supplemented with 10% (vol/vol) FBS and pen-step (Cellgro). HEK293TT cells [44] were cultured in DMEM supplemented with 10% (vol/vol) FBS, 1% Glutamax, 1% nonessential amino acids, and pen-strep (Invitrogen). Dicer wild-type cells (DLD1) and cells hypomorphic for Dicer activity (DLD1 DicerEx5−/−) cell lines were maintained in RPMI 1640 supplemented with 10% (vol/vol) FBS and pen-strep. Human B-cell line GM19240 was obtained from Coriell Institute and maintained in RPMI 1640 supplemented with 15% (vol/vol) FBS and pen-strep.

### Plasmids

Cassettes encompassing the predicted miRNA genes were synthesized by Integrated DNA Technologies (IDT) in the context of the pIDT-SMART-KAN vector (sequences are listed in Table S4). SV40 miRNA and MHV68 miRNA expression vectors have been previously described [12]. RISC Assay Luciferase reporters were generated with two long oligonucleotides of opposing orientations, which encoded for two complementary binding sites for the various miRNAs separated by eight nucleotides. Oligonucleotides were annealed and elongated using Taq polymerase (New England Biolabs) (98°C 30 s, 98°C 10 s, 55°C 20 s, 72°C 10 s,72°C 5 min). Extended target sites were then cloned into the XhoI/XbaI site pcDNA3.1dsRluc [39]. NMI wildtype and mutant 3′UTR reporters were synthesized as IDT gBlocks and subcloned into the XhoI/XbaI sites of pcDNA3.1dsRluc. pcDNA3.1dsRluc-GAPDH has been previously described [12].

### siRNAs and miRNA Mimics

TTV-tth8 miRNA mimics (pAGUAGUUGAGGCGGACGGUGGC, pCACCAUCAGCCACACCUACUCA) were synthesized by Sigma. Negative control si/miRNA mimic with Qiagen All Stars Negative Control sequence (pUUCUCCGAACGUGUCACGUdTdT, pACGUGACACGUUCGGAGAAdTdT) was synthesized by Sigma and has been described previously [45]. Drosha siRNA (pCGAGUAGGCUUCGUGACUUdTdT, pAAGUCACGAAGCCUACUCGdTdT) has been previously described [23]. NMI specific siRNAs (sc-36089) and negative control siRNA (sc-37007) were purchased from Santa Cruz Biotechnology.

### Generation of Lentiparticles

TTV-tth8 miRNA or an irrelevant miRNA (ebv-mir-BART4) was subcloned into the pLB2 CAG P2Gm (Addgene #19752) lentivector using XhoI and XbaI sites. The following plasmids were transfected into a T75 of HEK 293T cells using Lipofectamine 2000 (Invitrogen): 11.7 ug miR expression vector, 3.5 ug pMD2.G (Addgene #12259), 2.9 ug pRSV-Rev (Addgene #12253), and 5.9 ug pMDLg/pRRE (Addgene #12251). Supernatant was collected after 24 hours and the HEK293T cells were given fresh media. The next day, the supernatant was collected and combined with the previous day supernatant and 0.2 micron filtered. The stocks were titered on 10∧5 HEK293T cells in 24 well plates. Twenty microliters of serial dilutions of lentiparticle stocks were added to the cells in triplicate. After 48 hours, the cells were washed with PBS. Lentiparticle titers were determined by counting the percent of HEK293T cells that were GFP positive. Transducing units (TU) per mL was calculated using the following equation: ((Percent positive GFP×number of cells)/100× volume of viral dilution added to each well)×1/dilution factor.

### Generation of Stable Cell Lines Expressing TTV-tth8 miRNA

5×10∧5 GM19240 B-cells (Coriell Institute) were seeded into a 6-well plate. 1 mL of lentiparticles (1×10∧6 TU/mL) and 5 ul polybrene (Sigma-Aldrisch) (10 ug/mL) were added to each well in duplicate along with a polybrene only control. After 24 hours, the cells were pelleted and resuspended in fresh media along with puromycin (Sigma-Aldrich) (0.5 ug/mL). Cells were passed every 3 days in media that contained puromycin. The control B-cells did not survive past 2 passages with puromycin selection. After 17 days, selection was removed and cells were used for subsequent experiments.

### Generation of Recombinant Viruses

TTV-tth8 miRNA mutant virus plasmid (pUC-TTV-MUT) was generated by digestion of pUC-TTV-tth8 with AflII followed by treatment with mung bean nuclease (New England Biolabs) and self-ligation with T4 DNA ligase (New England Biolabs). The introduction of the expected 4 nt deletion was confirmed by sequencing. The pUC-TTV-SV40 miRNA virus plasmid was generated by PCR amplifying the miRNA encoding sequence of SV40-776 with primers PRIMER1, PRIMER2 and cloning into the AflII site of pUC-TTV-tth8. The introduction of the SV40 miRNA sequence in the same orientation as the wildtype miRNA was confirmed by sequencing.

### miRNA Prediction Software

Python scripts to predict pre-miRNA like structures in viral genomic sequence utilized the RNAfold [46] and Biopython [47] software packages. Scripts and associated data are freely available at https://code.google.com/p/mirna/

### Small RNA Northern Blots

Small RNA Northern blot analysis was performed as previously described [48]. Probe sequences are listed in Table S4.

### Preparation of Viral Genomes

Viral genome containing plasmids (150 ug) were digested with SalI-HF to release a linear viral genome sequence. Digests were heat inactivated and used to prepare dilute 30 mL T4 DNA ligase reactions. Ligations were incubated at 15C for 48 hours and then purified with HiPure Plasmid Maxiprep Kit (Invitrogen).

### Cell Culture Replication System

In vitro cell culture replication of TTV-tth8 and derivative viruses was carried out in HEK293TT cells transfected with viral genome preparations as previously described [15].

### DpnI Protection Assay

Genomic DNA was harvested by phenol/chloroform extraction [49]. Twenty micrograms of DNA was digested to completion with EcoRV-HF with or without DpnI. DpnI digest control was performed on twenty micrograms of DNA from pUC transfected HEK293TT cells spiked with 1 ng of TTV tth8 viral genome preparation. Southern blots were performed as described below [25].

### Southern Blots

Samples were run on 1% agarose TAE gels. Following electrophoresis, gels were soaked in 0.25 M HCL for 15 minutes. Next, gels were soaked in Southern Transfer Buffer (STB) (20 g/L NaOH, 87.5 g/L NaCl). Transfers to HyBond N+ membranes were performed overnight blot in STB. After transfer, membranes were soaked in neutralization buffer (100 mL Tris pH8, 50 mL 20× SSC, 350 mL H2O). Membranes were pre-hybridized for 1 hour at 60C in ExpressHyb Buffer (Clontech). Radiolabeled probes were generated using the Rediprime II DNA Labeling System (GE Healthcare) using SalI linearized TTV-tth8 genomic DNA. Probes were hybridized overnight at 60C. Blots were washed twice for 20 minutes with Wash Buffer 1 (2× SSC, 0.1% SDS) at 60C and twice for 20 minutes with Wash Buffer 2 (0.1× SSC, 0.1% SDS) at 50C. Storage phosphor screens (GE Healthcare) were exposed and then scanned using a Personal Molecular Imager system (Biorad).

### Synthetic Gene Small RNA Sequencing

Pooled, multiplexed small RNA sequencing was performed as previously described [12]. Genomic CDS maps were generated from the indicated reference sequence sequences with the Geneious software package (Biomatters).

### Cell Culture Replication System Small RNA Sequencing

HEK293TT cells were transfected with recircularized genome preparations or pUC control vector. Total RNA was harvested with PIG-B [50] at thirty hours posttransfection. Three hundred micrograms of total RNA was size fractionated on a 15% (vol/vol) UREA-PAGE gel and used to prepare small RNA libraries for Illumina small RNA sequencing. Sequencing adapter sequences were trimmed from the reads using custom Python scripts, and any sequences with ambiguous calls or less than 18 nt in length after trimming were removed from further analysis. The preprocessed reads were then mapped to the TTV-tth8 wt (AJ620231) or miRNA mutant genomic sequences using the SHRiMP2 software package [51]. 5′ start site counts and coverage were calculated using custom Python scripts and visualized using the gnuplot software package. Genomic CDS map was generated from the TTV-tth8 reference sequence with the Geneious software package (Biomatters).

### Analysis of In Vivo RNA Sequencing Data

SRA data files SRR039190 and SRR039191 were retrieved from NCBI. The SRA formatted files were converted to FASTA format and sequencing adapters were trimmed with custom Python scripts. The pre-processed files were mapped to a collection of TTV genomic sequences (Table S2) using the SHRiMP2 software package.

### Precursor miRNA Structure Prediction

miRNA stemloop secondary structures were generated using the Mfold RNA folding prediction Web server [52], [53] or the RNAfold prediction Web server [46], as indicated.

### RISC Activity Assay

Twelve well plates of HEK293 cells were co-transfected with five nanograms of *Renilla* luciferase based 3′UTR reporter (pcDNA3.1dsRluc [39]), five nanograms of firefly reporter (pcDNA3.1dsLuc2CP [39]) and one microgram of either empty vector (pIDT-SMART-KAN) or indicated TTV miRNA expression vector using the Turbofect reagent (Fermentas). Twenty-four hours later, cells were harvested and assayed with the Dual-Glo Luciferase Assay System (Promega). Luciferase activity was measured with a Luminoskan Ascent luminometer (Thermo Electronic). Student's t-test was used to assess statistical significance of observed differences.

### RNA Polymerase Activity Assay

HEK293 or HEK293T cells as indicated were transfected with viral genome preparations or miRNA expressions vectors. Two hours later, cells were treated with 50 ug/mL α-amanitin (Sigma). Total RNA was harvested with PIG-B [50] at 24 hours posttransfection and Northern blot analysis was performed.

### Drosha Dependence Assay

HEK293T cells were transfected with 20 nM Drosha siRNA or negative controls siRNA using Lipofectamine RNAi-MAX (Invitrogen). Twenty-four hours later, a second transfection of siRNA was performed followed by transfection of miRNA expression vectors using the Turbofect reagent according to the manufacturer's recommendations (Fermentas). Twenty-four or thirty hours later, total RNA was extracted with PIG-B and Northern blot analysis was performed.

### Dicer Dependence Assay

Dicer wild-type cells (DLD1) and cells hypomorphic for Dicer activity (DLD1 DicerEx5−/−) [24] were transfected with miRNA expression vectors using the Turbofect reagent (Fermentas). Twenty-four or thirty-six hours posttransfection, total RNA was extracted with PIG-B and Northern blot analysis was performed.

### Microarray Analysis

HEK293TT cells were transfected with recircularized genome preparations or pUC control vector [15]. One biological replicate was used for each treatment. Total RNA was harvested with PIG-B at thirty hours posttransfection. RNA was treated with DNase (Qiagen) and purified using RNeasy Minielute kit (Qiagen). RNA integrity was verified on a 1.0% agarose (Formaldehyde, MOPS) denaturing gel. The purified RNA was used as a template to make biotin labeled cRNA using an Illumina TotalPrep RNA Amplification Kit (Ambion) according to the manufacturer's guidelines. Labeled cRNA was precipitated overnight with isopropanol and sodium acetate. Biotinylated cRNA is hybridized to Illumina HumanHT-12 v4.0 BeadArray chips at the KECK Institute (Yale University) according to Illumina's protocols. Image analysis was carried out with BeadStudio software (Illumina) and initial quality controls (housekeeping genes, hybridization controls, and negative control probes) and data analysis (p-values for detection based on control probes and quantile normalization) were carried out with BeadStudio according to the instructions provided by Illumina. To identify candidate miRNA targets, the following criteria were applied: putative targets must be lower in the wildtype sample than the mutant or SV40 control and a seed complementary sequence must be present in the 3′UTR sequence of the candidate mRNA. Microarray data has been deposited in the GEO database. Candidate targets were then subject to subsequent validation assays as described in the Results section.

### Western Immunoblot Analysis

Fifty percent confluent six well plates of HeLa cells were transfected with 100 pmol of the indicated siRNA or miRNA mimic using Lipofectamine 2000 (Invitrogen). Forty-eight hours later, the transfected HeLa cells were split 1∶4. The next day, a second transfection was performed. Forty-eight hours later, lysates were prepared with RIPA buffer (0.1% SDS, 1% Triton X-100, 1% deoxycholate, 5 mM EDTA, 150 mM NaCl, and 10 mM Tris at pH 7.2) including Complete, Mini Protease Inhibitor tablets (Roche). Twenty micrograms of the total lysate was separated in 10% SDS-polyacrylamide gels and transferred to PVDF membranes (Millipore). Membranes were blocked with Odyssey blocking buffer (LI-COR). Primary antibodies used were Nmi (N-16): sc-9482 (Santa Cruz Biotechnology) and β-Actin (C4): sc-47778 (Santa Cruz Biotechnology). Blots were probed with a 1∶1000 dilution of each primary antibody in Odyssey blocking buffer. Blots were washed four times with Phosphate Buffered Saline including 0.1% Tween 20 (PBST). IRDye 800CW and IRDye 680LT secondary antibodies (LI-COR) were diluted 1∶10,000 in Odyssey blocking buffer containing 0.1% Tween 20 and 0.05% SDS. Blots were washed four times with PBST. Blots were scanned on an Odyssey CLx infrared imaging system (LI-COR). Band intensities were measured with Image Studio software (LI-COR). Three independent experiments were performed on different days for quantification and Student's t-test was used to assess statistical significance of observed differences.

### Interferon Signaling Assay

HEK 293T cells were seeded in 96-well plates. The next day, 1 ul Luciferase reporter mix (5 ng/ul pcDNA3.1dsRluc [39] and 20 ng/ul pISRE-Luc (Clonetech)) was co-transfected along with either RNA mimic (25 pmol/well), siRNA (25 pmol/well) or 100 ng re-circularized TTV genome. Mixed DNA/RNA transfections were performed with Lipofectamine 2000 (Invitrogen) and DNA only transfections were performed using the Turbofect transfection reagent according to the manufacturer protocol (Fermentas). In cases where both a miRNA mimic and siRNA were co-transfected, 25 pmol of both an RNA mimic and siRNA were used (50 pmol total) along with the Luc reporter mix. Each experimental condition was transfected into 6 wells (2 sets of triplicates-3 control wells and 3 experimental wells). After 48 hours, the media was replaced with new media with or without 100 u/ml of universal type I interferon (PBL Interferon Source). 16 hours after IFN treatment, a dual-luciferase assay was performed. Firefly luciferase was normalized to *Renilla* luciferase expression in order to control for transfection differences. Fold induction of the ISRE ffLuc reporter was calculated by dividing the comparable experimental wells by the control wells. Induction of each condition is relative to the negative control. Experiments with HeLa cells were conducted in a similar fashion except miRNA/siRNA transfections were performed in six well plates prior to seeding 96 well plates as described below. The HeLa cells were transfected with 50 pmol of siRNA or mimic (100 pmol for combined siRNA/miRNA transfection) using Lipofectamine 2000 (Invitrogen). Forty-eight hours later, cells were split 1∶4. The next day the cells were subject to a second round of transfection. Twenty four hours later, the HeLa cells were plated in 96 well plates. The next day, the interferon signaling assay was conducted as described above for HEK293T cells.

### Interferon Signaling Assay with Quantitative RT-PCR

HEK 293T cells in T25 plates were transfected with 7.5 ug plx304 plasmid (DNASU). Forty-eight hours later, the cells were replated in media containing 10 ug/mL Blasticidin S (Sigma-Aldrich). Antibiotic treatment was continued for four days and then removed for subsequent experiments. 12-well plates of HEK 293T were co-transfected with 40 ng pcDNA3.1dsRluc [39], 160 ng pISRE-Luc (Clonetech), and 80 pmol of the indicated siRNA or miRNA mimic using Lipofectamine 2000 (Invitrogen). Twenty-four hours later, the media was replaced with fresh media containing 100 units/ml of universal type I interferon (PBL Interferon Source). Sixteen hours after interferon treatment, total RNA was extracted using TRIzol Reagent (Invitrogen). Ten micrograms of total RNA was treated with one unit of DNAse I (NEB) for 30 minutes at 37C. DNAse treated RNA was ethanol precipitated. Two and a half micrograms of DNAse treated RNA was reverse transcribed using SuperScript III (Invitrogen) with oligo dT(20) primer (IDT). The cDNA was diluted to 100 ul. qPCR reactions consisted of 2 ul diluted cDNA, 1 ul (500 pmol) of each primer, 10 ul PerfeCta SYBR Green FastMix, ROX (Quanta Biosciences), and 6 ul water. ISG15 and GAPDH primers are listed in table S4. Real-time PCR program consisted of 2 minute incubation at 95°C followed by 40 cycles (15 s at 95°C, 30 s at 55°C, 15 s at 60°C). All qRT-PCR was performed on a StepOnePlus Real-Time PCR System (Applied Biosystems). Comparative Ct method was used with GAPDH serving as internal control gene for ISG15. Average relative quantities of three biological replicates each assayed in triplicate are reported.

### Interferon Growth Assay

3×10∧4 cells of the indicated pooled stable cell lines were seeded into a 6 well plate in 2 mL growth media in triplicate. Viable cells as assayed by trypan blue (Cellgro) staining were counted (Day 1) then 750 units universal type I interferon (IFN) (PBL Interferon Source) or 1 ug bovine serum albumin (BSA) (Sigma-Aldrich) control was added to the wells. Viable cell numbers were counted every day and after each cell count 750 units IFN or 1 ug BSA was added to the wells. Three independent experiments were performed on different days in triplicate.

## Supporting Information

Code S1 **miRNA Prediction Code.** Archive containing miRNA prediction code. Most recent version and additional files available at: https://code.google.com/p/mirna/.
(GZ) Click here for additional data file.

Figure S1 **TTV miRNAs expressed from synthetic vectors are generated by the canonical host miRNA biogenesis pathway.** (A) Northern blot analysis of RNA from HEK293T cells transfected with synthetic miRNA expression vectors with or without treatment with the RNA pol II inhibitor α-amanitin. Ethidium bromide stained low molecular weight RNA is shown as a load control. (B) Northern blot analysis of RNA from HEK293T cells co-transfected with synthetic miRNA expression vectors and either Drosha siRNA (siDrosha) or negative control siRNA (siNC). Ethidium bromide stained low molecular weight RNA is shown as a load control. (C) RISC reporter assay for synthetic TTV miRNA expression vectors. HEK293T cells were co-transfected with either empty miRNA expression vector (Vector) or indicated synthetic TTV miRNA expression vector and both firefly luciferase control and *Renilla* luciferase based reporter plasmids with vector UTR (Vector) or two sites perfectly complementary to the indicated miRNA. The average relative *Renilla* luciferase activity normalized to firefly luciferase activity of three replicates is shown. Error bars indicate SD of three replicates and p-values were calculated using Student's t-test.
(TIF)

Figure S2 **Characterization of cell culture genome replication of wildtype and miRNA mutant TTV-tth8.** Southern blot analysis of DpnI protection assay conducted on in vitro cell culture replication of wildtype TTV-tth8 (WT) and miRNA mutant TTV-tth8 (MUT). Lane NC is pUC transfected HEK293TT DNA and lane Ctrl is pUC transfected HEK293TT DNA spiked with viral genome prep. Replicated label indicates expected migration for linearized full length genomes. Input label indicates largest DpnI cleavage fragment.
(TIF)

Figure S3 **Knockdown of NMI by siRNA.** (A) Confirmation of siRNA mediated knockdown of NMI. Western blot analysis was performed on protein lysates from HeLa cells transfected with siRNA specific to NMI (siNMI) or negative control siRNA (siNC). (B) Interferon signaling assay performed in HeLa cells. Assay is performed as in Fig. 7C except HeLa cells were subjected to two rounds of mimic and siRNA transfection prior to plating for interferon signaling assay. Error bars indicate SD of three replicates and p-values were calculated using Student's t-test. Not significant (n.s.) indicates p-value greater than 0.05.
(TIF)

Table S1 **Pre-miRNA stemloop predictions for human TTVs and related animal viruses.**
(XLS)

Table S2 **Accessions for TTV genomic sequences used in small RNA sequencing analysis.**
(XLS)

Table S3 **Microarray analysis and list of putative TTV-tth8-miR-T1 targets.**
(XLSX)

Table S4 **Oligos and synthetic sequences used in this study.**
(XLS)
